The article "Combinatorial use of disulfide bridges and native sulfur-SAD phasing for rapid structure determination of coiled-coils" was published in 2018. Journal: Biosci Rep.

# Combinatorial use of disulfide bridges and native sulfur-SAD phasing for rapid structure determination of coiled-coils

**DOI:** 10.1042/BSR20181073

**Published:** 2018-09-19

**Authors:** Sebastian H.W. Kraatz, Sarah Bianchi, Michel O. Steinmetz

**Affiliations:** 1 Laboratory of Biomolecular Research, Division of Biology and Chemistry, Paul Scherrer Institut, CH-5232 Villigen PSI, Switzerland; 2 Biozentrum, University of Basel, CH-4056 Basel, Switzerland

**Keywords:** coiled-coil, disulfide bond, sulfur-SAD phasing, X-ray crystallography

## Abstract

Coiled-coils are ubiquitous protein–protein interaction motifs found in many eukaryotic proteins. The elongated, flexible and often irregular nature of coiled-coils together with their tendency to form fibrous arrangements in crystals imposes challenges on solving the phase problem by molecular replacement. Here, we report the successful combinatorial use of native and rational engineered disulfide bridges together with sulfur-SAD phasing as a powerful tool to stabilize and solve the structure of coiled-coil domains in a straightforward manner. Our study is a key example of how modern sulfur SAD combined with mutagenesis can help to advance and simplify the structural study of challenging coiled-coil domains by X-ray crystallography.

## Introduction

Coiled-coils are important protein–protein interaction motifs present in ∼3% of all eukaryotic proteins [1,2]. They consist of two or more amphipathic α-helices that wrap around each other’s hydrophobic seams resulting in parallel or antiparallel filamentous supercoils. Coiled-coils occur in many different types of proteins including ones of pathological relevance (e.g. they are implicated in cancer cell transformation and in Ebola virus–host interaction, respectively [3,4]). Although X-ray crystallography has classically been used to determine coiled-coil structures, difficulties in using this method are often encountered. The filamentous nature of coiled-coils can seriously hamper the crystallization process: while long coiled-coil fragments may interfere with the crystal formation, small constructs can prevent the folding into canonical coiled-coils resulting in unstable monomeric helices in solution or leading to incorrect assemblies due to the high protein concentration present in the crystal [5]. One way to overcome the length problem is to stabilize shorter coiled-coil fragments of interest under non-reducing conditions by cysteine crosslinking [6]. In addition to support crystallization, the presence of sulfur containing side chains bears further advantages for the subsequent structure determination process.

For coiled-coils, the inherent flexibility and possible heptad repeat discontinuities cause divergence from the canonical structure. This can result in a lack of suitable search models, which are required for successful molecular replacement [7,8]. Even recent adaptations of advanced computational methods tailored for coiled-coils [9,10] are limited by factors such as computational power, time and the availability of better than 2 Å resolution data. Therefore, experimental phasing is still an important method of choice for successful coiled-coil structure determination.

Due to the recent progress in detector and beamline technologies, native-SAD experiments can now be routinely performed and used for the *de novo* structure determination of protein crystals by X-ray crystallography [11–14]. By exploiting the native single-wavelength anomalous dispersion (SAD) of sulfur containing side chains, phasing can be achieved without the need for derivative datasets or selenomethionine-labeling. Here, we present a case study for the phase determination of coiled-coil structures using a combination of native or engineered cysteine crosslinking together with native SAD phasing. As test cases, we report two coiled-coil fragments that have been previously studied [15,16].

The first coiled-coil fragment is derived from CEP135, an important protein implicated in centriole formation. The two-stranded parallel coiled-coil fragment encompasses amino acids 82–144 of human CEP135 (referred to as HsCEP135 82–144) that contains one cysteine and one methionine per monomer. Notably, Cys110 of HsCEP135 82–144 is located in a heptad **d** core position and has been shown to be able to form a disulfide bridge in the context of its two-stranded parallel coiled-coil structure. The crystal structure of HsCEP135 82–144 has been recently solved by means of time and labor intense advanced molecular replacement approaches [15].

As a second case, we used the regulatory coiled-coil domain of the human kinesin-4 motor protein KIF21A. A recent study showed that the minimal KIF21A regulatory region folds into an intramolecular antiparallel coiled-coil monomer in solution, but crystallized into a dimeric domain-swapped antiparallel coiled-coil [16]. Here, we aimed to stabilize and crystallize the native, monomeric coiled-coil form of the KIF21A regulatory region by rationally introducing cysteine residues (the construct is hereafter referred to as Kif21a_M947C).

## Experimental procedures

### Protein production and purification

All constructs were generated to have a 6x-His-tag and a thrombin cleavage site using a positive selection cloning method [17]. The proteins were expressed in chemically competent BL21(DE3) cells (Stratagene) using LB media (50 μg/ml kanamycin and 30 μg/ml chloramphenicol for Kif21a_M947C and 50 μg/ml kanamycin for HsCEP135 82–144). Cells were grown to an OD_600_ of 0.6 at 37°C prior to induction with 0.5 mM isopropyl 1-thio-β-galactopyranoside (IPTG, Sigma-Aldrich). Protein expression was carried out at 20°C for ∼18 h. Cells were harvested by centrifugation. The cell pellets were resuspended in lysis buffer (HsCEP135 82–144: 50 mM HEPES, pH 8.0, 500 mM NaCl, 10 mM imidazole, 2 mM β-mercaptoethanol, 10 mM MgSO_4_ and one “cOmplete EDTA-free” protease inhibitor cocktail tablet (Roche Diagnostics); Kif21a_M947C: 50 mM HEPES, pH 8, 500 mM NaCl, 10 mM Imidazole, 10% glycerol and one “cOmplete EDTA-free” protease inhibitor cocktail tablet (Roche Diagnostics).

The resuspended cells were lysed on ice by ultrasonication. Lysate clearing was achieved by centrifugation for 30 min at 30000 rpm (105k ×***g***) in a Ti45 Rotor from Beckman Coulter, and the supernatant was filtered (0.45 µm filter). The filtrates were purified using a HiTrap Ni^2+^-Sepharose chelating column (Amersham) according to the manufacturer’s instructions. Following subsequent cleavage of the 6x-His-tag during dialysis overnight with thrombin (dialysis buffer: 20 mM Tris-HCl, pH 8.4, 150 mM NaCl and 2.5 mM CaCl_2_), a second affinity chromatography and a size-exclusion chromatography step (HiLoad Superdex 75 16/60, 20 mM Tris-HCl, pH 7.5, 150 mM NaCl) were performed. Purified protein samples were stored at −80°C until further use. The homogeneity of the recombinant proteins was assessed by SDS-PAGE and their identity was confirmed by ESI-TOF mass spectrometry.

### Biophysical analysis

Size-exclusion chromatography followed by multi-angle light scattering (SEC-MALS) experiments were performed in 20 mM Tris-HCl, pH 7.5, 150 mM NaCl, with or without 2 mM DTT using S-200 13/10 (M947C KIF21A) or 10/30 (HsCEP135 82–144) analytical size-exclusion chromatography columns (GE Healthcare) that were connected in-line to a mini-DAWN TREOS light scattering- and Optilab T-rEX refractive index detectors (Wyatt Technology). Protein samples were injected at the following volumes and concentrations: Kif21a_M947C, 100 μl at 2 mg/ml; HsCEP135 82–144 in the oxidized state, 100 μl at 4 mg/ml; HsCEP135 82–144 in the reduced state, 20 μl at 23 mg/ml.

Circular dichroism (CD) spectra were recorded at 5°C and at a protein concentration of 0.125 mg/ml in 1×PBS buffer supplemented with or without 5 mM TCEP or 2 mM DTT using a Chirascan spectropolarimeter (Applied Photophysics) and a cuvette of 0.1 cm path length. Thermal unfolding profiles between 5 and 90°C were recorded by increasing the temperature at a ramping rate of 1°C/min and monitoring the CD signal at 222 nm. Thermal melting temperatures were calculated using the Glob3 program (Applied Photophysics).

### Crystallization

HsCEP135 82–144 was crystallized at 20°C and at 15 mg/ml protein concentration using a condition from the Qiagen PACT screen (25% PEG 1500, SPG buffer, pH 6.0). No further cryo-protectant was required.

Kif21a_M947C was first crystallized at 20°C and at 18 mg/ml protein concentration using a commercial condition from the Qiagen pHClear screen (PEG 6000 30% 0.1 M citric acid, pH 4.0). The obtained crystals were subsequently crushed and used as a seed stock. Next, 200 nl of Kif21a_M947C at a concentration of 37 mg/ml were mixed at 20°C with 150 nl of mother solution of the Qiagen pHClearII screen together with 50 nl of the seed stock. Crystals for data collection grew in the Qiagen pHClearII screen condition 0.1 M HEPES, pH 7.0, 20% isopropanol and were soaked in 10% MPD as cryo-protectant.

### Data collection and processing

Data were collected at 100 K and at a wavelength of 2.0664 Å (as a trade of between maximizing the signal and minimizing the absorption; see [14]) at the beamline X60DA at the Swiss Light Source (Paul Scherrer Institut), which is equipped with a PRIGO multi axis goniometer and a Pilatus2M detector. The detector distance for data collection was 125.5 mm for Kif21a_M947C and 120.5 mm for HsCEP135 82–144, respectively. Data were collected at different chi angles. Further data collection parameters are given in Table 1. Per dataset 360° were collected at an exposure time of 0.1 s and an increment of 0.1° for Kif21a_M947C crystals, and at an exposure time of 1.0 s and an increment of 0.05° for HsCEP135 82–144 crystals.

**Table 1:** X-ray data collection and refinement statistics

Data collection	HsCEP135 82–144 PDB ID: 5NG4	Kif21aM947C PDB ID: 5NFD
Space group	I 41 22	P 21 21 21
Cell dimensions		
*a, b, c* (Å)	79 79 95.42	33.97 41.67 123.95
*α, β, γ*	90, 90, 90	90, 90, 90
Wavelength	2.07	2.07
Resolution (Å)	39.5–2.14 (2.21–2.14)	41.7–2.18 (2.25–2.18)
Chi angles	0°, 5°	20°
Total oscillation	2*360 °	1* 360°
*R*_merge_	0.089 (0.178)	0.031 (0.074)
*I*/σ	42 (7.2)	54.6 (9.6)
Completeness(%)	86 (43)	90 (35)
Redundancy	41.5 (6.2)	9.6 (2.1)
CC 1/2	0.999 (0.973)	1.0 (0.987)
Unique reflections	7467 (356)	8779 (336)
Refinement:		
Resolution (Å)	39.5–2.14	39.5–2.18
*R*_work_/*R*_free_	0.22/0.26	0.197/0.239
No. of atoms	946	1344
Protein	850	1244
Water	96	100
Average *B*-factors	47.0	34.5
Protein	47	34.6
Solvent	47.4	32.7
R.m.s. deviations		
Bonds length (Å)	0.001	0.002
Bond angles (°)	0.310	0.426
Ramachandran favored (%)	100	100
Ramachandran outliers (%)	0	0

Based on the preliminary data statistics resulting from the automated processing pipeline installed at the beamline, which is based on XDS and XSCALE [18], datasets were selected for further processing. Data reduction, integration and scaling were performed with the programs XDS and XSCALE [18]. In case of HsCEP135 82–144, data from two different chi angles (0° and 5°; Table 1) were merged. The scaled and merged data were converted into MTZ format using XDSCONV [19]. The *R*-free test dataset was generated using the reflection file editor from the PHENIX suite [20]. The fraction of reflection in the set was chosen to be 10% (PHENIX default value).

### Phasing

The structures were phased using SHELXC, SHELXD and SHELXE via the HKL2MAP interface [21,22]. Data up to 2.6 and 2.9 Å resolution were included into the heavy atom search for HsCEP135 82–144 and M947C KIF21A, respectively. This corresponded to a CC_1/2anom_ (self-correlation coefficient for the anomalous signal) of over 50% (Figure 3A, D ). Thousand trials were performed in SHELXD searching for 3 and 10 sulfide sites, respectively. The disulfide bridges were counted as one “super-sulfur” site. The resulting heavy atom substructures and derived phases were subjected to 20 cycles of density modification and model building with SHELXE. Based on the XTRIAGE analysis [20], the fractional solvent content was estimated at 0.52 and 0.48 for HsCEP135 82–144 and Kif21a_M947C, respectively.

The resulting phs files from the successful SHELXE tracing solutions were converted into the MTZ format using the phs2mtz script written out by hkl2map. The PHIM and FOM columns were combined with the MTZ file generated with XDSCONV [19] to produce the input MTZ file for BUCCANEER [23] using the reflection file editor from the PHENIX suite [20].

### Model building and refinement

The initial model was built with BUCCANEER [23] using the PHIM and FOM columns from the SHELXE output MTZ file for 20 cycles. The manual model building was carried out in COOT [24]. The model was refined with phenix.refine from the PHENIX suite [20]. Model-map correlations were calculated using the PHENIX suite. The refined structures were deposited in the Protein Data Bank (HsCEP135 82–144, PDB ID: 5NG4; Kif21a_M947C, PDB ID: 5NFD).

## Results

In the present study, we tested whether the combination of disulfide bridges as protein-stabilizing and -phasing tools aid the structure solution of challenging coiled-coil domains by X-ray crystallography. As test cases, we chose two coiled-coil protein fragments that have been previously studied [15,16]. Depending on the topology of the coiled-coil helices (e.g. arranged in a parallel or antiparallel manner), disulfide bridges can be introduced in heptad repeat positions that are forming the hydrophobic core of the coiled-coil. For certain positions, their Cα-Cβ bond vector positions them in close proximity to the core residue of the neighboring coiled-coil strand (neighboring **d** positions for parallel coiled-coils and neighboring **a** and **d** positions for antiparallel coiled-coils) [8]. In the first case, HsCEP135 82–144, we exploited the naturally occurring Cys110 located in a heptad **d** core position (Figure 1A), which has the ability to form a homotypic disulfide bond. In the second case, Kif21a_M947C, we recombinantly introduced a cysteine residue to stabilize and crystallize the native, monomeric coiled-coil from the KIF21A regulatory region. A schematic representation of the KIF21A intramolecular antiparallel coiled-coil (amino acids 938–1017) is provided in Figure 2A, illustrating that a native cysteine, Cys1006, is present in a heptad repeat **d c**ore position. We therefore introduced the cysteine mutation in the juxtaposed heptad acore position of the coiled-coil to allow for disulfide bridge formation.

**Figure 1:** Biophysical characterization of HsCEP135 82–144 (**A**) Amino acid sequence of HsCEP135 82–144. Heptad **a** and **d** positions are labeled with dark blue and light blue dots, respectively. (**B**) Far-ultraviolet CD spectra of HsCEP135 82–144 (20 μΜ) obtained at 5°C under oxidizing (gray) or reducing (blue) conditions. (**C**) Normalized thermal unfolding profiles of HsCEP135 82–144 obtained under oxidizing (gray) or reducing (blue) conditions recorded by CD at 222 nm. (**D**) Oligomerization state of HsCEP135 82–144 determined by SEC-MALS at 10°C under reducing (blue) or oxidizing (gray) conditions.

**Figure 2:** Biophysical characterization of the Kif21a_M947C (**A**) Model of the KIF21A intramolecular antiparallel coiled-coil. Heptad repeats are shown as blocks of seven residues with heptad core **a** and **d** positions indicated by dark blue and light blue dots, respectively. The predicted loop is shown in bold. The mutation M947C and the aspired cysteine crosslink are indicated in red. (**B**) Far-ultraviolet CD spectra of Kif21a_M947C (13 μM) obtained at 5°C under oxidizing (gray) or reducing (blue) conditions. (**C**) Normalized thermal unfolding profiles of Kif21a_M947C obtained under oxidizing (gray) or reducing (blue) conditions and recorded by CD at 222 nm. (**D**) Oligomerization state of Kif21a_M947C determined by SEC-MALS at 10°C.

### Biophysical characterization

In a first step, we performed a biophysical characterization of the two proteins under reducing and oxidizing conditions to evaluate the effect of the disulfide bridge on their fold and stability. The secondary structure content and the thermal stability were assessed by far-ultraviolet CD spectroscopy. As shown in Figure 1B, at 4°C and under reducing buffer conditions HsCEP135 82–144 (20 µM) revealed a CD spectrum characteristic of α-helical proteins with minima centered at 208 and 222 nm (Figure 1B). Thermal denaturation monitored by CD at 222 nm revealed a broad, non-cooperative unfolding profile typical of monomeric helices (Figure 1C) (Steinmetz et al., 2000; Steinmetz et al., 2001). These results suggest that under the conditions tried, HsCEP135 82–144 does not form a coiled-coil structure. However, under oxidizing conditions, promoting the formation of disulfide bridges, the recorded CD spectrum displayed characteristic features of α-helical coiled-coil proteins with a [Θ]_222_:[Θ]_208_ ratio of >1 [25] (Figure 1B). The thermal unfolding profile of HsCEP135 82–144 under oxidizing conditions revealed a cooperative unfolding profile (*T*_m_ of 62°C) characteristic of a well-folded protein (Figure 1C).

The CD spectra recorded for Kif21a_M947C under both reducing and oxidizing conditions revealed a significant amount of α-helical structure with distinct minima centered at 208 and 222 nm (Figure 2B). The stability of Kif21a_M947C was assessed by thermal unfolding profiles monitored by CD at 222 nm, which yielded a *T*_m_ value of 37°C under reducing and 69°C under oxidizing conditions (Figure 2C). These results indicate that Kif21a_M947C forms a well-folded protein under both reducing and oxidizing buffer conditions. However, the melting temperature under oxidizing conditions is drastically increased compared with reducing conditions, due to the engineered cysteine bridge.

To test the oligomerization state of both coiled-coils in solution, we performed SEC-MALS experiments. Under reducing conditions, we obtained a molecular mass of 9 kDa for HsCEP135 82–144, which is consistent with the presence of a monomer (calculated molecular weight of HsCEP135 82–144: 7.71 kDa). However, under oxidizing conditions a molecular weight corresponding to a dimer (16 kDa) was obtained (Figure 1D). As expected Kif21a_M947C was found to be monomeric under both reducing and oxidizing conditions (measured molecular mass: 11.3 kDa; calculated molecular mass: 9.5 kDa) (Figure 2D). We note that our SEC-MALS determined molecular masses for reduced HsCEP135 82–144 and Kif21a_M947C deviate from the calculated ones by 17 and 19%, respectively. This difference is most probably caused by the significantly reduced light scattering power of small proteins (<10 kDa) compared to larger ones.

Taken together, these results demonstrate that HsCEP135 82–144 only forms a two-stranded coiled-coil under oxidizing buffer conditions, while Kif21a_M947C forms a monomeric antiparallel coiled-coil structure under both reducing and oxidizing buffer conditions.

### Structure determination of HsCEP135 82–144

Data collection, processing and phasing for HsCEP135 82–144 were carried out as described in the ‘Experimental Procedures’ section following standard protocols (SigAno 2.33 in lowest resolution shell, anomalous correlation up to 2.39 Å; Table 1, Figure 3). The crystals diffracted to a higher resolution than it was possible to record with the detector at the chosen wavelength of 2.07 Å. Thus, resulting in a high *I*/sigma despite the limited completeness in the highest shell (see Table 1). The data analysis indicated two chains per asymmetric unit as the most probable composition (unit cell constants: 79 Å, 79 Å, 95.42 Å; 90°, 90°, 90°). Therefore, four sulfur atoms (two methionines and two cysteines) were expected, whereby the two cysteines were assumed to form a disulfide bridge based on the biophysical results (Figure 1). Consequently, the two cysteines were treated as one “super-sulfur” peak.

**Figure 3:** Anomalous sulfur phasing (**A**) and (**D**) Self-correlation coefficient of the anomalous signal as calculated by SHELXC for HsCEP135 82–144 (**A**, two datasets scaled together) and for Kif21a_M947C (**D**, one dataset), respectively. Resolution limits for phasing were chosen to yield a CC½ of >50% for the highest resolution. (**B**) and (**E**) CC_all_ versus CC_weak_ output for HSCEP135 82–144 (B) and Kif21a_M947C (**E**). (**C**) and (**F**) Plots showing contrast versus cycle for the density modification and chain tracing using the original hand (red) and the inverted hand (blue) for HsCEP135 82–144 (**C**) and for Kif21Acc M947C (**F**), respectively.

The heavy atom substructure search resulted in a cluster of distinct solutions that were separated from the main cluster with respect to CC_all_ versus CC_weak_ (Figure 3B). The subsequent density modification and automated chain tracing resulted in a CC of the partial structure against the native data of ~47% (starting from the inverted substructure phases). A clear gap between the solutions from the original and the inverted starting phases in the Contrast versus Cycle plot can be observed (Figure 3C). Ninety residues were built in three chains, indicating a clear solution.

Automated model building and refinement generated an initial model with a *R*_work_/*R*_free_ of 0.30/0.33. Further refinement and manual model building improved the *R*_work_/*R*_free_ to 0.22/0.26. The model-map cross-correlation between the initial map and the final model is 72.5%, indicating a high quality of the initial solution. The final structure contains two monomers in the asymmetric unit forming a two-stranded, parallel and in-register coiled-coil structure, consistent with the previous structure solved by molecular replacement [15]. A strong peak for the disulfide bridge formed by the cysteine residues at position 110 is visible in the anomalous difference map as well as the signal contributed by the methionines (Figure 4A). Though the protein construct ranged from amino acids 82–144 of HsCEP135, only residues 82–134 could be resolved. This is most likely due to an increased flexibility toward the termini of the coiled-coil. Together, these results demonstrate that it is possible to solve the structure of HsCEP135 82–144 in a fast and straight forward manner by sulfur-SAD using only two 360° degree datasets.

**Figure 4:** Structure of HsCEP135 82–144 (**A**) The HsCEP135 82–144 coiled-coil dimer as seen in the asymmetric unit of the crystal. The sulfur atoms are depicted as yellow spheres together with their anomalous difference density maps clipped at 3 σ (top) and with the 2Fo-Fc map at 1σ (bottom). (**B**) Two Kif21aM947C antiparallel coiled-coils constitute the asymmetric unit of the crystal. The sulfur atoms are depicted as yellow spheres together with their anomalous difference density maps clipped at 3 σ (top) and with the 2Fo-Fc map at 1σ (bottom). (**C**) Cartoon representation of chain B of the Kif21a_M947C structure. Heptad **a** and **d** positions as identified by SOCKET (26) are depicted in stick representation. Green, heptad **a** positions; orange, heptad **d** positions.

### Structure determination of Kif21a_M947C

The Kif21a_M947C coiled-coil fragment was crystallized under oxidizing buffer conditions. Data collection, phasing and refinement were carried out as described in the ‘Experimental Procedures’ section (see ’Experimental Procedures’ section, Table 1, Figure 3). For the purpose of phasing, a single dataset from the chi angle offset of 20° was chosen (Table 1) based on the anomalous signal strength (SigAno 3.048 in lowest resolution shell, anomalous correlation up to 2.51 Å). Data analysis indicated two monomers per asymmetric unit (unit cell constants: 33.97 Å, 41.67 Å, 123.95 Å; 90°, 90°, 90°), suggesting an overall count of 12 sulfur containing side chains. Cysteine bridges were treated as “super sulfurs”. The heavy atom substructure search resulted in a distinct cluster of solutions at high CC_all_/CC_weak_ separated from the main cluster of solutions (Figure 3E). Density modification resulted in a CC of 51.50% with 125 residues build in four chains indicating the correct solution, for the inverted substructure solution. The Contrast versus Cycle plot shows a clear gap between the original and inverted hand starting phases (Figure 3F).

Subsequent automated model building resulted in an initial model with a *R*_work_/*R*_free_ of 0.29/0.37. After further refinement and manual model building the final *R*_work_/*R*_free_ was reduced to 0.20/0.24. The overall model-map cross-correlation between the initial SHELXE map and the final model was 75%, illustrating the high quality of the initial solution. The final structure is composed of two intramolecular antiparallel coiled-coils per asymmetric unit with a disulfide bond between Cys947 and Cys1006 (Figure 4B). Clear peaks are visible in the anomalous difference map at positions of sulfur containing side chains (Figure 4B).

To assess whether the structure indeed follows the canonical coiled-coil heptad repeat pattern, we analyzed it with the program SOCKET [26]. The results revealed the classical knobs into holes packing mode with the pairing of heptad **a** and **d** positions forming **d/a** mixed layers typical of antiparallel coiled-coils [8] (Figure 4C). In conclusion, we solved the structure of an intramolecular antiparallel coiled-coil that is stabilized in its native conformation by a rationally introduced disulfide bridge.

## Discussion

Although many coiled-coil structures have been solved up to now and sophisticated coiled-coil prediction tools are available [27,28], the structure determination of coiled-coils by X-ray crystallography remains challenging [5,29]. Technical advances such as modern phasing softwares and detector technology now enable routine sulfur-SAD phasing experiments to be performed [13,30]. Benefiting from this development, our case study demonstrates that this phasing technique has matured to become a real alternative to the challenging procedures sometimes necessary to phase coiled-coils via molecular replacement methods. Especially in difficult cases, the chances of phasing coiled-coils may be significantly enhanced if anomalous sulfur datasets were to be collected. Our results clearly show that in favorable cases, two or even as few as one anomalous data set can be sufficient to phase a structure that otherwise would have been phased using more elaborate experimental or computational techniques as used in the previous studies of the investigated proteins [15,16]. In both cases presented herein the crystals diffracted beyond the resolution limit imposed by the chosen wavelength and beam line geometry. Reflections were recorded out to the very edge of the detector. As a result, the high quality diffraction of these crystals allowed collecting a strong *I*/sigma in the highest resolution shell (see Table 1). As expected, the higher number of sulfur containing side chains resulted in a higher anomalous signal for Kif21a_M947C. As with all experimental phasing techniques, sulfur-SAD benefits from a high crystal quality. In case of less well diffracting crystals, sulfur-SAD should be combined with other phasing techniques to improve the overall chances of success.

The increased stability obtained by exploiting disulfide bridges [6,31] allows for the generation of a higher diversity of coiled-coil fragments of a given protein, which can be screened for successful crystallization. Coiled-coils are especially suitable for the rational introduction of disulfide bridges and our approach can easily be applied *ab initio* as a variety of algorithms are available, which predict the heptad repeat pattern with high accuracy [27,32–34]. Depending on the coiled-coil topology (parallel or antiparallel) cysteine mutations can be introduced at the juxtaposed **d** and **d’** and **a** and **d’** positions, respectively. The application of this protein engineering principle not only allowed us to stabilize an otherwise monomeric coiled-coil fragment in its native dimeric structure, but also to crystallize an antiparallel monomeric coiled-coil in its native conformation. To the best of our knowledge, only one crystal structure of an antiparallel monomeric coiled-coil in isolation has been published so far in the Protein Data Bank [35], highlighting the advantage of our approach. In conclusion, our case study shows that cysteine crosslinking and phasing via sulfur-SAD is a particular useful strategy to solve coiled-coil structures by X-ray crystallography. It benefits from straightforward prediction of suitable mutation sites to introduce disulfide bridges and it can be easily combined with other phasing strategies [36,37].

## Abbreviations

HsCEP135: human centrosomal protein of 135 kDa
KIF21a: kinesin-like protein KIF21A
MALS: multi-angle light scattering
Sulfur-SAD: Sulfur-single-wavelength anomalous dispersion
